This article has been retracted.

# Effect of Autologous Stem Cell Transplantation Combined with Modified VTD Regimen on Elderly Patients with Multiple Myeloma and Its Influence on miRNA Cytokines

**DOI:** 10.1155/2022/6320329

**Published:** 2022-02-16

**Authors:** Zhaoliang Bai, Jiansong Shen

**Affiliations:** ^1^Outpatient Department, 971 Hospital of the Chinese People's Liberation Army Navy, Qingdao, Shandong 266000, China; ^2^Department of Rehabilitation Medicine and Physiotherapy, 971 Hospital of the Chinese People's Liberation Army Navy, Qingdao, Shandong 266000, China

## Abstract

**Objective:**

To explore the effect of autologous stem cell transplantation combined with modified VTD regimen on elderly patients with multiple myeloma and its influence on miRNA cytokines.

**Methods:**

The data of 42 elderly patients with multiple myeloma who were treated in our hospital from May 2010 to June 2018 were retrospectively analyzed, and they were divided into the combined group (autologous stem cell transplantation combined with improved VTD scheme, *n* = 25) and the control group (improved VTD scheme, *n* = 17) according to different treatment schemes, and the clinical efficacy of the two groups was compared. The levels of CD3+, CD4+, CD4+/CD8+, and Treg were measured in the two groups. The expression levels of miRNA-15a, miRNA-16, and miRNA-21 in the bone marrow fluid of the two groups were measured before and after treatment. The levels of M protein and myeloma cells in the two groups were detected. Comparing the incidence of adverse reactions between the two groups, the Kaplan-Meier method was used for survival analysis.

**Results:**

The total effective rate of the combined group (84.00%) was higher than that of the control group (52.94%), and the difference was statistically significant (*P* < 0.05). After treatment, the levels of CD3+, CD4+, CD4+/CD8+, Treg, miRNA-15a, and miRNA-16 in the combined group were higher than those in the control group, and the levels of miRNA-21, M protein, and myeloma cells were lower than those in the control group, with statistical significance (*P* < 0.05). There was no significant difference in adverse reactions between the two groups (*P* > 0.05). The first, second, and third year survival rates of group A (96.00%, 88.00%, and 80.00%) were significantly higher than those of the control group (70.59%, 58.82%, and 47.06%), and the difference was statistically significant (*P* < 0.05).

**Conclusion:**

Autologous stem cell transplantation combined with a modified VTD regimen can effectively improve the immune function and survival rate of elderly patients with multiple myeloma, which is safe and effective.

## 1. Introduction

Multiple myeloma (MM) is a common malignant tumor in the blood system, the incidence rate of which accounts for 1% of all tumors and 15% of all tumors in the blood system, and it is mostly found in elderly men over 65 years old [1, 2]. The cause of the disease is unknown. Its clinical features are malignant proliferation of clonal plasma cells and secretion of tumor protein-M protein, which damages various organs of the body. Typical clinical manifestations are renal insufficiency, anemia, hypercalcemia, and bone destruction [3, 4]. At present, the clinical treatment of MM mostly adopts traditional chemotherapy, new targeted therapy, and hematopoietic stem cell transplantation (HSCT). In the traditional era of chemotherapy, the total response rate of multiple myeloma patients to chemotherapy was less than 50% [5, 6]. In recent years, the research and development of some new drugs and the development of treatment technology have effectively improved the survival time and quality of life of patients [7, 8]. Bortezomib, as a new protease inhibitor, is effective in the treatment of multiple myeloma, and it is recommended as the first-line drug for the treatment of myeloma [9, 10]. The traditional VTD regimen is bortezomib+thalidomide+dexamethasone, in which thalidomide is a glutamic acid derivative, which can inhibit angiogenesis, regulate immunity, and resist tumor. Dexamethasone is a glucocorticoid drug, which has anti-inflammatory and immunosuppressive effects. Bortezomib combined with thalidomide and dexamethasone can alleviate drug resistance, but the traditional VTD regimen is easy to cause adverse reactions such as peripheral neuropathy. It has been shown that the incidence of peripheral neuropathy can be reduced by adjusting the dose and mode of administration of bortezomib to ensure the overall efficiency. Therefore, this study adjusted the single dose of bortezomib administration based on the previous study [11]. Autologous hematopoietic stem cell transplantation (auto-HSCT) collects autologous hematopoietic stem cells before pretreatment, stores them in vitro, and then transfuses them after patients receive radiotherapy and chemotherapy, so as to rebuild the immune function and hematopoietic function. In addition, autologous hematopoietic stem cell transplantation can effectively prolong the survival time of patients with multiple myeloma, because there is no donor source limitation, and the transplant mortality of patients is low.

MicroRNA (miRNA) refers to a kind of noncoding single-stranded RNA with a length of 21~25 nt, which can combine with mRNA 3 noncoding region to degrade or inhibit translation and regulate the process of cell apoptosis, differentiation, and proliferation. As a noncoding small molecule RNA, it can directly degrade target genes and can posttranscriptionally regulate genes. According to related studies, abnormal miRNA expression can be closely related to the proliferation, differentiation, and apoptosis of multiple myeloma cells, and some miRNAs can be used as effective targets for the treatment of MM [12]. The change of miRNA expression level can be used to monitor the progress of multiple myelom, and can also be used as a marker for diagnosis of multiple myeloma. At present, some studies have shown that miRNA-21 is closely related to the occurrence, invasion, metastasis, and drug resistance of tumors, and some studies have taken miRNA as a gene therapy target for multiple myeloma [11–13]. Many patients with multiple myeloma have immune dysfunction, and their gene subtypes and chromosomal abnormalities are related to certain miRNAs, and more than 50% of miRNAs are located in genomic regions such as amplification region, cleavage site, fragile site, and loss of heterozygosity. miRNA is closely related to the immune regulation and differentiation function of the adaptive immune system. It is considered that miRNA-15a and miRNA-16 are closely related to multiple myeloma in academic circles. According to relevant studies, miRNA-15a and miRNA-16 levels are abnormally expressed in multiple myeloma cell lines, and bortezomib can upregulate the expression levels of miRNA-15a and miRNA-16 [14]. The purpose of this study is to explore the effect of autologous stem cell transplantation combined with a modified VTD regimen on elderly patients with multiple myeloma and its influence on miRNA cytokines, which is reported as follows.

## 2. Data and Methods

### 2.1. General Data

The data of 42 elderly patients with multiple myeloma treated in our hospital from May 2010 to June 2018 were retrospectively analyzed. According to different treatment schemes, they were divided into the combined group and control group, 25 cases in the combined group and 17 cases in the control group. There were 14 males and 11 females in the combined group. The average age was 69.32 ± 5.00 years. Myeloma types are as follows: IgG type in 11 cases, IgA type in 8 cases, and light chain type in 6 cases; ISS (International Staging System) is as follows: stage I 6 cases and stage IIA 7 cases; stage IIIA: 8 cases; and stage IIIB: 4 cases. There were 10 males and 7 females in the control group. The age ranged from 61 to 77 years, with an average of 68.71 ± 4.06 years. Myeloma types are as follows: IgG type in 7 cases, IgA type in 5 cases, light chain type in 5 cases; ISS (International Staging System): 4 cases in stage I, 5 cases in stage IIA. There were 4 cases of stage IIIa and 4 cases of stage IIIB. The general data of the two groups were compared (*P* > 0.05). The study was approved by the hospital ethics committee (approval no. 2020-SYYDK-023), and the patients and their families gave informed consent to the study (see Table 1).

### 2.2. Inclusion Criteria

Inclusion criteria were as follows: (1) All patients were diagnosed as multiple myeloma by clinical pathological diagnosis. (2) All of them meet the diagnostic criteria of multiple myeloma [15], serum M protein ≥30 g/l and/or bone marrow clonal plasma cells ≥ 10%, accompanied by any of the following symptoms: hypercalcemia (>11.5 mg/l or 2.65 mmol/l), renal insufficiency (serum creatinine > 2 mg/dl or >177 μmol/l), anemia (hemoglobin < 10 g/dl or <normal level 2 g/dl), combined with a pathological fracture or osteolytic destruction and other bone diseases. (3) 60 years old ≤ age ≤ 80 years old. (4) The combined group was assessed to be suitable for autologous stem cell transplantation and modified VTD regimen, while the control group was assessed to be suitable for a modified VTD regimen. (5) Meet the indications of autologous stem cell transplantation. (6) Complete clinical case data.

### 2.3. Exclusion Criteria

Exclusion criteria were as follows: (1) Patients with a clear diagnosis of MM according to the revised diagnostic criteria of the international myeloma working group (IMWG) in 2020 [16]. (2) Those with poor compliance. (3) Those who are allergic to the drugs used in this study. (4) Patients with other malignant tumor diseases. (5) Patients with severe infectious diseases.

### 2.4. Methods

The control group was treated with modified VTD. Bortezomib (Xi'an Janssen Pharmaceutical Co., Ltd., gyzz: j20160071) 1.6 mg/m^2^ was injected intravenously on the 1st, 8th, and 15th days. Thalidomide (Changzhou Pharmaceutical Factory Co., Ltd., national drug approval: h32026129) 100~200 mg/d was given orally before going to bed. Dexamethasone (Sinopharm Rongsheng Pharmaceutical Co., Ltd., Sinopharm Junzi: h41020036) 20~40 mg/d was given intravenously on the 1st~ 2nd, 8th~ 9th and 15th~ 16th days. One course of treatment was 28 days and four courses of treatment. The combined group was treated with autologous stem cell transplantation combined with improved VTD scheme. The combined group received autologous stem cell transplantation after 4 courses of modified VTD treatment. First, 4 ~ 5.25 g/m^2^ cyclophosphamide chemotherapy was used (Baxter Oncology GmbH, import drug registration number: H20160467), coupled with hematopoietic growth factor mobilization. On the 8th day, recombinant human granulocyte colony-stimulating factor (rhGCSF) was used for routine mobilization until the end of collection. CD34+ cells were collected by CS3000plus blood cell separator with a content > 2 × 10^6^/kg, and CD34+ cells were (2.12~ 37) detected by flow cytometry ×10^6^/kg and store it in liquid nitrogen at - 196°C. Two days before transplantation, high-dose melphalan was injected intravenously for pretreatment, with a standard of 200 mg/m^2^. On the day of transplantation, APSC was reinfused, with a content of 248~ 804 ml and a mononuclear cell volume (MNC) of (2.43 ~ 38.3) × 10^8^/kg, CD34+ cells (2.12 ~ 37) × 10^6^/kg. Cell transplantation was performed in laminar flow ward, anti-infection treatment and red blood cell infusion were appropriately performed, and rhG CSF 5 UG/kg/d was injected subcutaneously. The content of leukocytes which was more than >1.0 × 10^9^/l was transferred to the general ward.

### 2.5. Observation Indexes

(1) Clinical efficacy: the two clinical outcomes were assessed according to the International Myeloma Working Group and classified as complete remission (CR), very good partial remission (VGPR), partial remission (PR), stable disease (SD), and progressive disease (PD). (2) Immunological function: the levels of CD3+, CD4+, CD4+/CD8+, and Treg in the two groups were measured by flow cytometry. (3) miRNA cytokine level: the expression levels of miRNA-15a, miRNA-16, and miRNA-21 in the bone marrow fluid of the two groups before and after treatment were measured by real-time fluorescence quantitative PCR (RT-PCR), and miRNA primer design was obtained by querying the Sanger microRNA sequence database, which is difficult to design, but reverse transcription of microRNA into cDNA was used for detection. The designed primers are as follows: miRNA-15a: forward primer 5′-CGCCTAGCAGCACACATAATGG-3′; miRNA-16: forward primer 5′-GCCGTAGCAGCACGTAAATA-3′; and miRNA-21: forward primer 5′-GTGCAGGGTCCGAGGT-3′. (4) The levels of M protein and myeloma cells in the two groups were detected by automatic biochemical analyzer. (5) Adverse reactions such as neutropenia, infection, thrombocytopenia, fatigue, anemia, gastrointestinal reactions, thrombosis, cardiotoxicity, peripheral neuropathy, and hepatic and renal impairment. Those were judged according to the international standard of unified nomenclature for toxic and side effects of tumor tissues NCICTCAE [17]. (6) Analysis of survival curve: the follow-up methods of discharge from hospital are telephone, outpatient, etc. The follow-up frequency is once a month in the first year, once a month in the second year, and once a month in the third year. The survival time of the two groups is recorded, and the Kaplan-Meier method is used to analyze the survival situation of the two groups.

### 2.6. Evaluation Criteria of Curative Effect

According to the international myeloma working group (IMWG) [18], the clinical curative effects of the two groups were evaluated, which were divided into complete remission (CR), excellent partial remission (VGPR), partial remission (PR), disease stability (SD), and disease progression (PD). CR: hematuria was negative by immunofixation electrophoresis, the ratio of bone marrow plasma cells was less than or equal to 5%, and soft tissue plasma cell tumor disappeared. VGPR: on the basis of satisfying CR condition, sFLC △ ratio is normal, and no clonal plasma cells were found in the bone marrow by flow cytometry. PR: if hematuria M protein can be measured, the blood M protein will decrease by ≥50% and urine M protein < 200 mg/24 hours or decrease by ≥90%. If the hematuria M protein is not detected, the difference between sFLC and sFLC will be reduced by ≥50%.If sFLC and hematuria M protein are not measurable, the proportion of bone marrow plasma cells will be reduced by ≥50%, the proportion of bone marrow plasma cells will be ≥30% in the baseline period, and the volume of soft tissue plasma cell tumor will be reduced by ≥50% in the baseline period. SD: none of them meet the above standards. PD: urine M protein level increased by ≥25% compared with the baseline value. If hematuria M protein is unmeasurable, it is required that the difference between sFLC and sFLC should be 10 mg/dl, bone marrow plasma cells should be increased by 10%, or new bone destruction or soft tissue plasma cell tumor or original volume should be increased. Total effective rate (ORR) = (CR + VGPR + PR)/total cases × 100%.

### 2.7. Statistical Methods

SPSS 20.0 statistical software was used to analyze and process the data, and the measurement data was expressed as *x* ± *s*. Independent sample *T* test was used for comparison between groups, paired *T* test was used for comparison before and after treatment within groups, and the counting data was expressed as frequency and composition ratio, and test *χ*^2^ or Fisher accurate probability test was used. The Kaplan-Meier method was used to analyze the survival situation of the two groups, and *P* < 0.05 suggested that the difference was statistically significant.

## 3. Results

### 3.1. Comparison of Clinical Efficacy between the Two Groups

There were 21 patients in the combined group who achieved treatment effectiveness and 9 patients in the control group. The total effective rate of the combined group was 84.00% and that of the control group was 52.94%. The overall efficiency of treatment was higher in the combined group than in the control group, and the difference between the two groups was statistically significant (*P* < 0.05) (see Table 2).

### 3.2. Comparison of Immune Function before Treatment

There was no significant difference in CD3+, CD4+, CD4+/CD8+, and Treg levels between the two groups (*P* > 0.05). After treatment, the levels of CD3+, CD4+, and CD4+/CD8+ in both groups increased, and the levels of CD3+, CD4+, CD4+/CD8+, and Treg in the combined group were higher than those in the control group, and the differences were statistically significant (*P* < 0.05) (see Table 3).

### 3.3. Comparison of miRNA Cytokine Levels between the Two Groups

Before treatment, there was no significant difference in miRNA-15a, miRNA-16, and miRNA-21 levels between the two groups (*P* > 0.05). After treatment, the levels of miRNA-15a and miRNA-16 increased and the level of miRNA-21 decreased in the two groups. The levels of miRNA-15a and miRNA-16 in the combined group were higher than those in the control group, and the level of miRNA-21 was lower than that in the control group, with statistical significance (*P* < 0.05) (see Table 4).

### 3.4. Comparison of M Protein and Myeloma Cell Levels between the Two Groups

Before treatment, there was no significant difference in M protein and myeloma cell levels between the two groups (*P* > 0.05). After treatment, the levels of M protein and myeloma cells in both groups decreased, which was significantly lower in the combined group than in the control group (*P* < 0.05) (see Table 5).

### 3.5. Adverse Reactions in Both Groups Included Neutropenia, Infection, Thrombocytopenia, Fatigue, Anemia, Gastrointestinal Reactions, Thrombosis, Cardiotoxicity, Peripheral Neuropathy, and Hepatic and Renal Impairment, with no Statistically Significant Differences (*P* > 0.05) (See Table 6)

### 3.6. Comparison of Survival Time between Two Groups

The survival rates in the first, second, and third years of follow-up in the combined group (96.00%, 88.00%, and 80.00%) were significantly higher than those in the control group (70.59%, 58.82%, and 47.06%) (*P* < 0.05) (see Table 7, Figures 1–3).

## 4. Discussion

Multiple myeloma is a common blood system disease in the elderly, but the traditional chemotherapy method has no significant effect on this disease. Bortezomib is a new reversible inhibitor of chymotrypsin-like activity of 26S proteasome. Bortezomib can promote the apoptosis of tumor cells by transplanting the tumor signal transduction pathway and can increase the sensitivity of radiotherapy [16, 19].VTD regimen can effectively regulate the body's immunity, improve the microenvironment of the bone marrow, promote the apoptosis of tumor cells, etc. It can effectively prolong the patients' survival time and improve their quality of life. However, some patients have serious adverse reactions during the treatment and cannot continue the treatment, among which peripheral neuropathy becomes a common adverse reaction, and patients can show numbness of their hands or feet, which seriously affects their quality of life. According to related studies, the incidence of peripheral neuropathy can be reduced by changing the administration method, dose, and cycle of bortezomib [20, 21], and the dose and cycle of bortezomib were changed by the improved VTD protocol in this study. Autologous stem cell transplantation collects autologous hematopoietic stem cells in vitro before pretreatment and then transfuses them after patients receive ultrahigh-dose radiotherapy and chemotherapy pretreatment, which is helpful to rebuild hematopoietic function and immune function. The treatment of multiple myeloma has the advantages of safety, effectiveness, and few complications. NCCN guidelines clearly indicate that autologous hematopoietic stem cell transplantation has become the first-line treatment scheme suitable for patients with multiple myeloma. At present, autologous stem cell transplantation has been widely used in the treatment of patients under 65 years old [22, 23]. In this study, autologous stem cell transplantation combined with modified VTD scheme was applied to the treatment of elderly patients with multiple myeloma, in order to explore the best clinical treatment scheme for elderly patients with multiple myeloma.

In this study, after treatment, the total effective rate (84.00%) of the combined group was significantly higher than that of the control group (52.94%), and after treatment, the levels of CD3+, CD4+, CD4+/CD8+, and Treg in the combined group were higher than those in the control group, indicating that the combined scheme is effective in treating elderly multiple myeloma and can effectively improve the immune function of patients. Bortezomib in the improved VTD scheme is an artificial protease inhibitor, which can effectively destroy the adhesion of myeloma cells, hydrolyze specific proteins, inhibit the expression of growth factors and genes of myeloma cells, and promote the apoptosis of myeloma cells. In addition, bortezomib can effectively relieve the immune suppression microenvironment, reduce the tumor load of patients, and improve the immune function. There are also clinical studies that the combination of bortezomib-containing chemotherapy and autologous stem cell transplantation can effectively improve the therapeutic effect [24]. The improvement of immune function in the combination group is better than that in the control group, which may be because autologous stem cell transplantation is helpful to rebuild hematopoietic function and immune function. M protein is an abnormal immunoglobulin produced by plasma cells or B lymphocytes, while myeloma cells are caused by abnormal plasma cell proliferation [25]. In this study, after treatment, the improvement degree of M protein and myeloma levels in the combined group is better than that in the control group, indicating that the combined treatment of elderly multiple myeloma can more effectively improve the body's immunity and inhibit the proliferation of myeloma cells.

According to related studies, the expression levels of miRNA-15a, miRNA-16, and miRNA-21 are closely related to patients' responsiveness to chemotherapy drugs, which can be used to predict the prognosis of patients. miRNA-15a and miRNA-16 can show abnormal expression in multiple myeloma cell lines. Clinically, the growth and proliferation of multiple myeloma cells can be inhibited by adjusting the levels of miRNA-15a and miRNA-16. miRNA-15a, miRNA-16, and miRNA-21 are related to the level of serum tumor burden markers. miRNA-21 is the main driving force of miRNA transcription, closely related to the growth, invasion, and metastasis of tumors, and abnormally expressed in various tumor tissues. According to related studies, the level of miRNA-21 in the refractory group of multiple myeloma patients is higher than that in the remission group or control group, and the levels of miRNA-15a and miRNA-16 are lower than that in the remission group or control group [26]. In this study, the levels of miRNA-15a and miRNA-16 in the combined group are higher than those in the control group, and the level of miRNA-21 is lower than that in the control group, which indicates that the patients in the combined group have a higher degree of remission and the combined scheme has a better effect in treating elderly multiple myeloma. There was no significant difference in the incidence of adverse reactions between the two groups, which indicated that although the combined scheme increased the treatment means, it did not increase the adverse reactions, which indicated that autologous stem cell transplantation was safe. Serious adverse reactions can occur during conventional VTD treatment. In the present study, the combined regimen did not increase the incidence of adverse reactions despite the additional treatment. This suggests that the safety of the treatment is guaranteed while improving its effectiveness. It can increase patient compliance and better implementation [27]. Compared with the control group (70.59%, 58.82%, and 47.06%), the survival rates in the first, second, and third years of follow-up in the combined group were significantly higher than those in the control group (96.00%, 88.00%, and 80.00%), which indicated that the combined regimen could effectively prolong the survival time of patients with multiple myeloma and improve their survival rates. It has also been shown in previous studies that the combination regimen was well tolerated by patients and significantly improved survival [28].

To sum up, this study combined autologous stem cell transplantation with a modified VTD protocol compared to the traditional VTD protocol. Autologous stem cell transplantation combined with modified VTD regimen is effective in the treatment of patients with multiple myeloma, which can effectively improve their immune function and enhance their survival rate, with good safety and clinical application value. For patients who were suitable for autologous stem cell transplantation, clinicians may consider a combined VTD regimen to improve patient prognosis. The deficiency of this study lies in the need for autologous stem cell transplantation, strict inclusion criteria, fewer cases included in the study, and the number of cases can be increased for further research.

## Figures and Tables

**Figure 1:** Survival curve of combined group and control group for one year.

**Figure 2:** Survival curve of combined group and control group for two years.

**Figure 3:** Survival curve of the combined group and control group during a 3-year follow-up.

**Table 1:** Comparison of general data between the two groups.

	Combined group (*n* = 25)	Control group (*n* = 17)	*χ* ^2^/P
Male/female(case)	14/11	10/7	0.325
Age(years)	69.32 ± 5.00	68.71 ± 4.06	0.068
Myeloma types IgG/IgA/light chain (case)	11/8/6	7/5/5	0.765
ISS (International Staging) stage I/stage IIA/stage IIIA/stage IIIB (case)	6/7/8/4	4/5/4/4	0.059

**Table 2:** Comparison of clinical efficacy between two groups (cases (%)).

Groups	CR	VGPR	PR	SD	PD	ORR
Joint group (*n* = 25)	8 (32.00)	6 (24.00)	7 (28.00)	2 (8.00)	2 (8.00)	21 (84.00)
Control group (*n* = 17)	2 (11.76)	3 (17.65)	4 (23.53)	3 (17.65)	5 (29.41)	9 (52.94)
*χ* ^2^ *value*						4.783
*P* value						0.029

**Table 3:** Comparison of immune function between two groups (*x* ± *s*, *%*).

Group	CD3+		CD4+		CD4+/CD8+		Treg	
	Before treatment	After treatment	Before treatment	After treatment	Before treatment	After treatment	Before treatment	After treatment
Joint group (*n* = 25)	57.29 + 5.74	67.94 + 5.63^a^	31.29 + 3.10	43.36 + 3.21a	0.99 + 0.30	1.69 + 0.25a	3.19 + 0.67	4.69 + 0.88a
Control group (*n* = 17)	55.06 + 4.48	59.90 + 2.99^a^	30.03 + 1.35	34.56 + 2.76^a^	1.03 + 0.16	1.23 + 0.17^a^	3.31 + 1.02	4.02 + 1.03
*T* value	1.344	5.381	1.566	8.186	0.376	5.774	0.476	2.257
*P* value	0.187	<0.001	0.125	<0.001	0.709	<0.001	0.637	0.030

Note: compared with the same group before treatment, ^a^*P* < 0.05.

**Table 4:** Comparison of miRNA cytokine levels between two groups (*x* ± *s*).

Group	miRNA-15a		miRNA-16		miRNA-21	
	Before treatment	After treatment	Before treatment	After treatment	Before treatment	After treatment
Joint group (*n* = 25)	1.05 + 0.35	2.75 + 0.26^a^	1.14 + 0.47	2.76 + 0.21^a^	3.45 + 0.57	2.33 + 0.39^a^
Control group (*n* = 17)	1.09 + 0.29	2.01 + 0.39^a^	1.14 + 0.36	1.98 + 0.21^a^	3.70 + 0.86	2.74 + 0.46^a^
*T* value	0.329	7.377	0.036	11.918	1.126	3.117
*P* value	0.744	<0.001	0.971	<0.001	0.267	0.003

Note: compared with the same group before treatment, ^a^*P* < 0.05.

**Table 5:** Comparison of M protein and myeloma cell levels between two groups (*x* ± *s*).

Group	M protein (g/l)		Myeloma cell (×10-2 *μ*g/ml)	
	Before treatment	After treatment	Before treatment	After treatment
Joint group (*n* = 25)	54.52 + 4.35	23.37 + 1.73a	35.55 + 3.86	15.91 + 1.37^a^
Control group (*n* = 17)	53.08 + 5.25	34.56 + 3.82a	34.73 + 2.93	23.28 + 2.48^a^
*T* value	0.966	12.867	0.745	12.388
*P* value	0.340	<0.001	0.461	<0.001

Note: compared with the same group before treatment, ^a^*P* < 0.05.

**Table 6:** Comparison of adverse reactions between the two groups (cases (%)).

Group	Neutropenia	Infected	Thrombocytopenia	Fatigue asthenia	Anemia	Gastro intestinal reaction	Thrombus	Cardio toxicity	Peripheral neuropathy	Liver and kidney dysfunction
Joint group (*n* = 25)	3 (12.00)	2 (8.00)	2 (8.00)	17 (68.00)	5 (20.00)	22 (88.00)	5 (20.00)	1 (4. 00)	7 (28.00)	1 (4. 00)
Control group (*n* = 17)	2 (11.76)	2 (11.76)	1 (5.88)	11 (64.71)	3 (17.65)	13 (76.47)	2 (11.76)	1 (5. 88)	2 (11.76)	0 (0. 00)
*χ* ^2^ value	0.001	0.166	0.068	0.049	0.036	0.968	—	—	1.584	—
*P* value /Fisher value	0.982	0.683	0.794	0.824	0.849	0.325	0.681	1.000	0.208	1.000

**Table 7:** Comparison of survival time between two groups (cases (%)).

Group	Follow-up 1 year		Follow-up for 2 years		Follow-up for 3 years	
	Survive	Die	Survive	Die	Survive	Die
Joint group (*n* = 25)	24 (96.00)	1 (4.00)	22 (88.00)	3 (12.00)	20 (80.00)	5 (20.00)
Control group (*n* = 17)	12 (70.59)	5 (29.41)	10 (58.82)	7 (41.18)	8 (47.06)	Yy (52.94)
Log-rank *χ*^2^ value	5.267		5.112		5.649	
*P* value	0.022		0.024		0.018	

## Data Availability

The labeled dataset used to support the findings of this study is available from the corresponding author upon request.
